The article "The Promotional Effect of Hollow MnO2 with Brucea Javanica Oil Emulsion (BJOE) on Endometrial Cancer Apoptosis" was retracted in 2024. Reasons: signs of a paper mill; compromised peer review; unreliable results or conclusions.

# The Promotional Effect of Hollow MnO_2_ with Brucea Javanica Oil Emulsion (BJOE) on Endometrial Cancer Apoptosis

**DOI:** 10.1155/2021/6631533

**Published:** 2021-03-18

**Authors:** Qin Hu, Shu Zhang, Jun Zhu, Lina Yin, Suping Liu, Xiaowei Huang, Guihao Ke

**Affiliations:** Department of Gynecology, Fudan University Shanghai Cancer Center, Shanghai, China

## Abstract

Endometrial cancer (EC) is a common gynecological malignancy worldwide whose therapy mainly depends on chemotherapy. In past years, an increasing number of studies indicate that hollow MnO_2_ could serve as a nanoplatform in the drug delivery system. The Brucea javanica oil emulsion (BJOE) has been illustrated to play a vital role in cancers. However, knowledge about the combined effect of H-MnO_2_-PEG/BJOE in endometrial cancer remains ambiguous up to now. In the present work, we prepared a drug-delivery vector H-MnO_2_-PEG by chemical synthesis and found that H-MnO_2_-PEG significantly inhibited cell proliferation in endometrial cancer cells. Moreover, the combination of H-MnO_2_-PEG/BJOE could repress cell proliferation more efficiently and promote cell apoptosis. Mechanistically, we found that BJOE exerted its role as a promoter of endometrial apoptosis by regulating relative protein expressions. In general, the present study demonstrates that H-MnO_2_-PEG functions as a critical vector in the tumor microenvironment of endometrial cancer and the significant effect of H-MnO_2_-PEG/BJOE on cancer cells, suggesting a new paradigm for the treatment of endometrial cancer.

## 1. Background

Nowadays, endometrial cancer is the most common reproductive cancer in women, and the introductory presentation of which is abnormal uterine bleeding [1]. Type I endometrial cancer is estrogen-dependent and represents 75-90% of endometrial cancer, while type II endometrial cancer is estrogen independent [2–4]. Histopathological examination of the endometrial biopsy specimen and endometrial cytological examination of the endometrial brush is the leading diagnoses. 320,000 women are diagnosed with endometrial cancer each year, and there are 76,000 mortalities associated with endometrial cancer worldwide [5–8]. The rate of endometrial cancer (EC) is steadily increasing so far, and the current treatment remains chemotherapeutics, which may result in menopausal symptoms. Therefore, new and more efficient therapeutic methods need to be explored for this disease.

Although chemotherapy has been extensively employed in the clinic, the therapeutic efficacy may be dramatically restricted by nonspecific drug release and severe side effects [9]. With the swift development of nanotechnology [10–12], the application of various nanomaterials for cancer nanomedicine has drawn wide attention in recent years [13–16]. Compared with traditional chemotherapeutic drugs, nanoanticancer drug therapy has potential application prospects in curing cancer diseases. One of the significant concerns about nanoanticancer drugs is the drug-delivery vector.

In recent years, nanodrug delivery system has developed rapidly. Yang et al. [17] reported the synthesis and functionalization of monodisperse hollow structured MnO2 (H-MnO2) and further verified their protective effect on ischemic stroke. Lately, manganese oxide (MnO_2_) nanostructures are treated as a unique type of tumor microenvironment-responsive nanocarrier for cancer theranostics. For instance, Fan et al. presented that MnO_2_ could interact with acidic H_2_O_2_ to generate sufficient oxygen in the tumor microenvironment, thereby promoting the efficacy of hyperoxia-dependent radiophotodynamic therapy [18]. Besides, MnO_2_ could react with intracellular GSH, which led to the mitigation of high GSH levels for more efficient photodynamic treatment. Previous studies also confirmed that Mn ions could improve the T1-weighted magnetic resonance (MR) imaging contrast for tumor-specific imaging and detection [19–21]. By contrast, the structure of hollow MnO_2_ has been proposed to be a predominant nanocarrier to load many therapeutic agents, with the releasing behavior in response to the specific tumor microenvironment. However, the therapeutic efficacy of HMnO_2_ on endometrial cancer remains elusive, and, therefore, studies are needed to explain such association.

For the synthesis of hollow MnO_2_ (H-MnO_2_) that underlies the drug delivery system, the solid SiO_2_ nanoparticles are widely used as hard templates, and the resulting H-MnO_2_ takes on orderly morphology and is highly monodisperse. Afterward, the high surface area and mesoporous shells of as-prepared H-MnO_2_ take shape, and finally, the H-MnO_2_ is electrostatically coated with diamine polyethylene glycol (PEG). In the current study, we set experiments to explore the function of H-MnO_2_-PEG and the Brucea javanica oil emulsion (BJOE), traditional Chinese medicine that is of great use to kill cancer cells [22], on endometrial cancer cells, especially investigating its effects on cell proliferation and apoptosis.

## 2. Materials and Methods

### 2.1. Materials

Polyallylamine hydrochloride (PAH, MW ~15,000) and polyacrylic acid (PAA, MW ~1800) were commercially supplied by Sigma-Aldrich. Triton-X 100, 1-octanol, NaOH, Ammonia aqueous solution (28 wt %), and tetraethyl orthosilicate (TEOS) were purchased from Aladdin Industrial Inc. (Shanghai, China). Diamine-ploy (ethylene glycol) (Mw ~2000) was provided by JenKem Technology Co. Ltd. (Beijing, China). A dialysis bag with a molecular weight cut-off (MWCO) of 3.5 kDa was ordered from Spectrum Inc. Co. Ltd. (Shanghai, China). All other chemicals were purchased from Sinopharm, Inc. Co. Ltd. (Shanghai, China) and used as received. Deionized (DI) water was used throughout the experiments. All glassware was washed with aqua regia and then rinsed with ethanol and DI water before use.

### 2.2. Synthesis and Modification of H-MnO_2_ Nanoparticles

The solid SiO_2_ nanoparticles were synthesized by a modified Stöber method [22]. Typically, 6 mL of TEOS was added to a solution containing 72 mL of ethanol, 8 mL of deionized water, and 1.5 mL of ammonia aqueous, stirring for 8 h, and the products were collected by centrifugation and washed by water and ethanol for several times. The obtained samples were dried in a vacuum at 40°C for 8 h. Then, 100 mg SiO_2_ nanoparticles and 0.2 g MnCl_2_•4H_2_O were mixed with 50 mL of water by sonication for 15 min. After that, 0.5 g urea was added, and the mixture was stirred in an oil bath at 90°C for 2 h. The products were collected by centrifugation and washed by water and ethanol. The products were calculated at 600°C. Then, the silica template was removed by using 0.5 M NaOH (50°C for 24 h). The obtained H- MnO_2_ was collected by centrifugation and washed by water and ethanol. The prepared H-MnO_2_-PEG was obtained by centrifugation and washed with water for three times. Finally, to conjugate FA onto H-MnO2-PEG, 10 mg of FA was dissolved in 10 mL of DMSO containing 6.3 mg EDC and 4.7 mg NHS. After stirred for 3 h, 50 mg of H-MnO_2_-PEG was added and treated for 12 h.

### 2.3. Characterization

The morphology of prepared samples was observed using JEOL-1400 transmission electron microscopy (TEM) at 120 kV. Scanning electron microscopy (SEM) images were performed with a Hitachi S-4800 ultrahigh-resolution cold FEG with an in-lens electron optic operating at 20 kV.

### 2.4. Cell Culture

Human endometrial cancer cells (RL95-2) were obtained from American Type Culture Collection (ATCC). RL95-2 cells were cultured in DMEM/F12 supplemented with 10% FBS and 1% PSN, in an atmosphere of 5% CO_2_ at 37°C.

### 2.5. Cell Viability

Cell Counting Kit-8 (CCK-8) assay was carried out to detect RL95-2 cell viability with CCK-8 reagent (Takara, Japan). The cells were plated at 5 × 10^3^ cells/well into 96-well plates and treated with BJOE, H-MnO_2_-PEG, or H-MnO_2_-PEG/BJOE for 48 h. After that, the cells were incubated with 10 *μ*L CCK-8 for another 2 h at 37°C. The absorbance was measured at 450 nm with a microplate reader (Bio-Rad, Hercules, CA, USA).

### 2.6. Flow Cytometry

An annexin V-FITC/PI Apoptosis Detection Kit (Sigma-Aldrich, St. Louis, MO, USA) was used to determine the apoptotic rate of cells as per the manufacturer's instructions. Briefly, RL95-2 cells treated with BJOE, H-MnO_2_-PEG, or H-MnO_2_-PEG/BJOE for 48 h were washed with precooled culture medium twice, centrifuged at 2000 rpm for 5 min to collect cells (3 × 10^5^), and then suspended with 500 *μ*l binding buffer (culture medium with magnesium, calcium, 0.5% NaN3, and 1% FBS). Thereupon, Annexin V (5 *μ*l), and PI (10 *μ*l) were added to the cells and incubated for 10 min at room temperature in the dark. A flow cytometer (Attune NxT; Thermo Fisher Scientific, Inc.) and ModFitLT software were used to detect and calculate the percentage of apoptotic cells.

### 2.7. Western Blot

The total protein from RL95-2 cells was extracted and homogenized in RIPA buffer (Sigma-Aldrich). The concentrations of the extracted nuclear and cytoplasmic fractions were quantified using the bicinchoninic acid assay (BCA) method. A total of 30 *μ*g protein per sample was separated by SDS-PAGE (12%) and then transferred to a PVDF membrane, prior to blocking with 5% nonfat milk in 1xTBST, overnight at 4°C. The membrane was then incubated with anti-Caspase-3 (1 : 1000; ab32351; Abcam), anti-KRas (1 : 1000; ab275876; Abcam), anti-Raf1 (1 : 1000; ab236003; Abcam), anti-ERK1/2 (1 : 1000; ab184699; Abcam), anti-p-ERK1/2 (1 : 1000; ab223500; Abcam), and anti-GAPDH (1 : 10000; ab181602; Abcam) primary antibodies overnight at 4°C. After washing 3 times in 1xTBST, the membranes were incubated with the corresponding HRP-conjugated secondary antibody (1 : 5000; ab205718; Abcam) for 1 h at room temperature. The immunoreactive proteins were visualized by an enhanced chemiluminescence reaction, and the band density was calculated by ChemiDoc™ XRS+ Imaging system (Bio-Rad).

### 2.8. Statistical Analysis

The data was expressed as mean ± standard deviation (SD) and analyzed by one-way analysis of variance (ANOVA). ^∗^*p* < 0.05 and ^∗∗^*p* < 0.01 indicate a statistical difference between the parallel groups.

## 3. Results

### 3.1. Synthesis and Characterization of H-MnO_2_-PEG

The synthetic procedure of H-MnO_2_-PEG is shown in Figure 1. First, MnO_2_ was deposited onto solid SiO_2_ nanoparticles in situ, and then the hollow-structured MnO_2_ nanomaterials were formed by etching the solid SiO_2_. For functionalization of the H-MnO_2_, the diamine polyethylene glycol (PEG) was coated onto the negative surface of H-MnO_2_ by electrostatic assembly later, thus, the H-MnO_2_-PEG was synthesized to deliver the drug for endometrial cancer more efficiently.

Next, we carefully characterized the obtained nanoparticles. As shown in Figure 2, transmission electron microscope (TEM) images showed that solid SiO_2_ nanoparticles were uniformly spherical with an average particle diameter of about 150 nm (right), which could also be found in scanning electron microscopic (SEM) images in different magnifications (left).

### 3.2. The Repressive Effect of H-MnO_2_-PEG on Cancer Cell Proliferation

Given that nano-MnO2 serves as a unique nanocarrier responsive to tumor microenvironment for cancer therapy and hollow MnO2 structure is regarded as the main nanocarrier that can load a large amount of therapeutic drugs, we further explore the therapeutic effect of H-MNO2-PEG on endometrial cancer. To explore the monotherapy of H-MnO_2_-PEG, we measured the intensity of endometrial cancer cells (RL95-2) in different concentration gradients (0 *μ*g/mL, 25 *μ*g/mL, and 50 *μ*g/mL) of the synthesized nanomaterials. As shown in Figure 3(a), the intensity gradually decreased as the concentration increased, suggesting that H-MnO_2_-PEG served as an inhibitor to the proliferation of endometrial cancer cells. Such obtained results the first time uncovered the correlation between H-MnO_2_-PEG nanoplatform and endometrial cancer, which provided a significant prospect of a novel treatment for the severe carcinoma of the endometrium.

### 3.3. Combination of H-MnO_2_-PEG/BJOE Inhibits Cell Proliferation More Effectively

As uncovered in the previous study, BJOE could regulate the relative tumor genes to kill cancer cells directly [22–25]. Besides, it had also been verified to repress the resistance reaction of tumor cells to chemotherapy and significantly improve body immunity [26]. To further understand the function of BJOE on endometrial cancer cells, the cellular activity of RL95-2 was observed for 48 h after the single BJOE (50 *μ*g/mL), the single H-MnO_2_-PEG, or the combination of H-MnO_2_-PEG/BJOE by CCK-8 assay and DAPI assay. It was found that both the cellular activity and cell number declined in both the H-MNO2-PEG group and H-MNO2-PEG/BJOE group compared with the BJOE treatment group (Figures 3(b) and 3(c)). Moreover, the combination of H-MnO_2_-PEG/BJOE had shown better efficacy in inhibiting cancer cell proliferation, which reveals a more effective medicinal effect of the combination of H-MnO_2_-PEG/BJOE on killing the endometrial cancer cells.

### 3.4. Combination of H-MnO_2_-PEG/BJOE Promotes Apoptosis of Endometrial Cancer

We next explored the effect of H-MnO2-PEG/BJOE on apoptosis of endometrial carcinoma cells. Flow cytometry results showed that H-MnO_2_-PEG significantly increased the apoptosis of endometrial cancer cells, while H-MnO2-PEG/BJOE further promoted the apoptosis of endometrial carcinoma cells (Figure 4). Additionally, western blot assay showed that H-MnO2-PEG/BJOE significantly enhanced the expression level of Caspase-3, KRas, and Raf1, compared with the only H-MnO_2_-PEG group (Figure 5). Taken together, the results indicated that H-MnO_2_-PEG/BJOE could efficiently suppress tumor growth and enhance cell apoptosis by modulating the expression of relative genes.

## 4. Discussion

Rational utilization of the characteristics of tumor microenvironment and development of responsive nanoscale drug delivery system for tumor microenvironment can achieve targeted drug delivery and controlled release in tumor sites, reduce toxic side effects of chemotherapeutic drugs, and improve drug efficacy. The utilization of nanoparticle-based drug delivery approaches to treat cancer cells has played a vital role in overcoming the limitations of traditional therapeutic approaches [27]. For instance, it was illustrated that the application of a carbohydrate coated iron oxide nanoparticle-ferumoxytol (FDA approved) as an iron supplement has been widespread for curing several diseases like chronic kidney disease, IDA, and cancer [28–30]. As depicted in the results, our developed H-MnO_2_-PEG nanoplatform with efficient tumor-homing capacity could effectively release the chemotherapeutic drug upon responsive to tumor acidic microenvironment with respect to endometrial cancer.

In recent years, Chinese medicine has gradually become a good choice for treating various forms of cancers and the improvement of the disease symptoms, especially for BJOE therapy. The previous study showed the effects of BJOE combined with transcatheter hepatic arterial chemoembolization (TACE) on primary liver cancer (PLC) and the related mechanisms [22]. Moreover, injection of BJOE has been widely used for lung cancer (LC) in China, which is known to provide favorable outcomes with conventional treatments [31]. In the current study, we have fabricated hollow mesoporous MnO_2_ nanoshells with PEG coating as a multifunctional theranostic platform responsive to endometrial cancer and repress cell proliferation and compared the effect of individual H-MnO_2_-PEG and the combination of H-MnO_2_-PEG/BJOE. Further combination of H-MnO_2_-PEG/BJOE offers a more eminent effect to inhibit the growth of endometrial cancer cells. Subsequent experiments demonstrate that this combinational therapy strategy would enhance tumor apoptosis mainly by modulating relative proteins' expression. With inherent biodegradability, our H-MnO_2_-based theranostic nanoplatform may indeed find significant potential in clinical translation to allow the combination of chemotherapy and cancer immunotherapy, which could offer a comprehensive synergistic effect in battling cancer.

## 5. Conclusion

In conclusion, we successfully synthesized the highly monodispersed hollow MnO2 with a mesoporous shell and applied it as an effective nanocarrier for targeting chemotherapy of endometrial cancer. The structure of H-MnO_2_-PEG developed here was confirmed by TEM images, and the nanoparticle presented a specific advantage in suppressing the cell proliferation of endometrial cancer. Besides, the combination of H-MnO_2_-PEG/BJOE demonstrated the killing effect of BJOE on cancer cells and tumor inhibition efficacy. Moreover, BJOE could promote apoptosis in endometrial cancer by regulating protein expressions. Overall, the present study offered a novel paradigm of the MnO2-based drug delivery system to exert endometrial cancer treatment.

## Figures and Tables

**Figure 1:** Schematic illustration of the synthesis process of H-MnO2-PEG.

**Figure 2:** Structural characterizations of H-MnO2-PEG. (a) Representative SEM images of H-MnO2-PEG. Scale bars = 200 nm. (b) Representative TEM images of H-MnO2-PEG. Scale bars = 100 nm. SEM: scanning electron microscope; TEM: transmission electron microscope; H-MnO2-PEG: hollow MnO_2_-PEG.

**Figure 3:** Combination of H-MnO_2_-PEG/BJOE inhibits RL95-2 cell proliferation more effectively. (a) The intensity of endometrial cancer cells (RL95-2) was measured with different concentrations of H-MnO_2_-PEG (0 *μ*g/mL, 25 *μ*g/mL, 50 *μ*g/mL) treatment by DAPI staining. (b) The cell activity of RL95-2 was detected after BJOE (50 *μ*g/mL), H-MnO_2_-PEG, or H-MnO_2_-PEG/BJOE combination treatment for different times (0, 12, 24, and 48 h) by CCK-8 assay. (c) The cell proliferation of RL95-2 was detected after BJOE (50 *μ*g/mL), H-MnO_2_-PEG, or H-MnO_2_-PEG/BJOE combination treatment for 48 h by DAPI staining. DAPI: 2-(4-Amidinophenyl)-6-indolecarbamidine dihydrochloride; BJOE: Brucea javanica oil emulsion; H-MnO_2_-PEG: hollow MnO_2_-PEG. ^∗^*p* < 0.05, ^∗∗^*p* < 0.01, ^∗∗∗^*p* < 0.001.

**Figure 4:** Combination of H-MnO_2_-PEG/BJOE promotes RL95-2 cell apoptosis more effectively by flow cytometry. The cell apoptosis of RL95-2 was detected after BJOE (50 *μ*g/mL), H-MnO_2_-PEG, or H-MnO_2_-PEG/BJOE combination treatment for 48 h by flow cytometry. BJOE: Brucea javanica oil emulsion; H-MnO_2_-PEG: hollow MnO_2_-PEG.

**Figure 5:** Combination of H-MnO_2_-PEG/BJOE promotes RL95-2 cell apoptosis more effectively by western blot. Western Blot analysis for Caspase-3, KRas, Raf1, p-ERK1/2, and ERK1/2 protein expression level in RL95-2 cells treated with BJOE (50 *μ*g/mL), H-MnO_2_-PEG, or H-MnO_2_-PEG/BJOE combination. BJOE: Brucea javanica oil emulsion; H-MnO_2_-PEG: hollow MnO_2_-PEG; p-ERK1/2: ERK1/2 phosphorylation.

## Data Availability

Some or all data, models, or codes generated or used during the study are available from the corresponding author by request.
